# Mechanism of *Radix Astragali* and *Radix Salviae Miltiorrhizae* Ameliorates Hypertensive Renal Damage

**DOI:** 10.1155/2021/5598351

**Published:** 2021-04-21

**Authors:** Guangjian Hou, Yuehua Jiang, Yuekun Zheng, Meng Zhao, Yuanzhen Chen, Yonghao Ren, Congan Wang, Wei Li

**Affiliations:** ^1^Neck-Shoulder and Lumbocrural Pain Hospital of Shandong First Medical University, Jinan 250062, China; ^2^Central Laboratory, Affiliated Hospital of Shandong University of Traditional Chinese Medicine, Jinan 250011, China; ^3^Rizhao Traditional Chinese Medicine Hospital, Rizhao 276826, China; ^4^Department of Nephrology, Affiliated Hospital of Shandong University of Traditional Chinese Medicine, Jinan 250011, China

## Abstract

Hypertensive-induced renal damage (HRD) is an important public health and socioeconomic problem worldwide. The herb pair *Radix Astragali*- (RA-) *Radix Salviae Miltiorrhizae* (RS) is a common prescribed herbal formula for the treatment of HRD. However, the underlying mechanisms are unclear. The purpose of our study is to explore the mechanism of combination of *Radix Astragali* (RA) and *Radix Salviae Miltiorrhizae* (RS) ameliorating HRD by regulation of the renal sympathetic nerve. Thirty 24-week-old spontaneously hypertensive rats (SHRs) as the experimental group were randomly divided into the RA group, the RS group, the RA+RS group, the valsartan group, and the SHR group and six age-matched Wistar Kyoto rats (WKY) as the control group. After 4 weeks of corresponding drug administration, venipuncture was done to collect blood and prepare serum for analysis. A color Doppler ultrasound diagnostic instrument was used to observe renal hemodynamics. Enzyme-linked immunosorbent assay was used to detect norepinephrine (NE), epinephrine (E), angiotensin II (Ang II), and B-type brain natriuretic peptide (BNP). Simultaneously, the kidneys were removed immediately and observed under a transmission electron microscope to observe the ultrastructural changes. And the concentration of transforming growth factor-*β*1 (TGF-*β*1), angiotensin type 1 receptor (AT1), and nitric oxide (NO) was detected by immunohistochemistry. Our results showed that renal ultrasonography of rats showed no significant difference in renal size among groups. The RA+RS group had obviously decreased vascular resistance index. The levels of NE, E, BNP, Ang II, AT1, and TGF-*β*1 were decreased (*P* < 0.05), and the density of NO was increased. Pathological damage of the kidney was alleviated. In conclusion, the results of the present study suggested sympathetic overexpression in the pathogenesis of HRD. The combination of RA and RS may inhibit the hyperexcitability of sympathetic nerves and maintain the normal physiological structure and function of kidney tissue and has a protective effect on the cardiovascular system.

## 1. Introduction

Hypertensive-induced renal damage (HRD) is a critical reason of end-stage renal disease [1]. Among the causes of end-stage renal disease, HRD accounts for nearly 34% of the total number of cases [2]. Studies have shown that the progression of HRD is closely related to renal sympathetic nerve hyperexcitability [3]. Renal sympathetic nerve hyperexcitability affects HRD patients mainly in three aspects, including changes in blood pressure, progression of kidney disease, and cardiovascular complications [3, 4]. Sympathetic nerve hyperexcitability can lead to increased volume load, cause abnormal activation of RAS, ultimately increase blood pressure, and promote cardiovascular complications [5]. In addition, sympathetic nerve excitement directly acts on the kidneys, causing blood pressure to rise [6].

In traditional Chinese medicine, “invigorating qi and promoting blood circulation” is currently one of the most widely used treatments for hypertensive kidney damage. *Radix Astragali* (RA, Huangqi in Chinese) and *Radix Salviae Miltiorrhizae* (RS, Danshen in Chinese) are the most commonly used compatibility drugs. In our previous research, we focused on investigating the role of traditional Chinese medicine in chronic kidney disease. Studies have shown that RA is commonly used for treating nephrotic syndrome [7]. RA is used in large amounts and can reduce blood pressure, increase renal nitric oxide level, improve the expression of NOS, scavenge oxygen free radicals, and block the oxidation reaction. To protect the structural and functional integrity of renal vascular and improve vascular endothelial function [8], RS exhibits multiple pharmacological activities such as vasorelaxation, antioxidation, and antiapoptotic effects in renal cells [9].

Based on the above understanding, the research on the efficacy of RA and RS against chronic kidney disease is relatively clear. However, the pharmacological effects of RA and RS on hypertensive kidney injury are still unclear. Therefore, this study is aimed at investigating the effects of herb pair RA and RS in spontaneously hypertensive rats (SHRs) and determining the underlying mechanism by regulation of the renal sympathetic nerve.

## 2. Materials and Methods

### 2.1. Animals and Experimental Methods

Thirty 17-week-old male SHRs and six age-matched Wistar Kyoto rats (WKY) were obtained from Beijing Weitong Lihua Experimental Animal Technology Co., Ltd., China (No. SCXK (Beijing) 2012-0001). They were fed in the Experiment Animal Center of Affiliated Hospital of Shandong University of Traditional Chinese Medicine. All procedures of the project were approved by the Faculty of Medicine and Health Sciences Ethics Committee for Animal Research, Affiliated Hospital of Shandong University of Traditional Chinese Medicine.

Studies have shown that SHR kidney damage occurs at an average age of 6 months, so after feed with food and water for 2 months. The random number table is divided into the RA group, the RS group, the RA+RS group, the valsartan group (used as positive control), the SHR group, and the WKY group. The SHR group and the WKY group were intragastrically administered with saline. SHRs in other groups (RA group, RS group, RA+RS group, and valsartan group) were intragastrically administered the corresponding drugs once daily for 28 days. The blood pressure was recorded at 7-day interval.

### 2.2. Renal Ultrasonography and Tissue Collection

The renal ultrasonography was performed on small animals under anesthesia with sodium pentobarbital (30 mg/kg, intraperitoneal injection) using a color Doppler ultrasound diagnostic instrument (M5Vet, Mindray, China) [10]. Computer software (M5Vet) was used to record and analyze renal hemodynamics.

After 4 weeks of drug administration, the rats were euthanized with intraperitoneal injection of sodium pentobarbital (40 mg/kg). Venipuncture was done to collect blood and prepare serum for analysis. Enzyme-linked immunosorbent assay (ELISA) was used to detect norepinephrine (NE), epinephrine (E), angiotensin II (Ang II), and B-type brain natriuretic peptide (BNP). Simultaneously, the kidneys were removed immediately, one part was fixed with 4% paraformaldehyde, and the concentration of transforming growth factor-*β*1 (TGF-*β*1), angiotensin type 1 receptor (AT1), and nitric oxide (NO) was detected by immunohistochemistry (IHC). In the second part, the ultrastructure changes were observed under a transmission electron microscope (TEM, JEOL 1200EX, Electron Optics Laboratory Co. Ltd., Japan). The remaining tissues were homogenized for western blot assay.

### 2.3. IHC Staining of TGF-*β*1, AT1, and NO in Rat Renal Tissue

Renal sections were stained with rabbit anti-rat TGF-*β*1, AT1, and NO (Abcam, 1 : 150 dilution, China; Ab92486, Ab18801, and Ab66127) at 4°C overnight. Then, sections were incubated with horseradish peroxidase- (HRP-) conjugated AffiniPure goat anti-rabbit IgG (ZSGB-Bio, ZB-2301, 1 : 100, China) at room temperature for 60 min [10]. Tissue sections were colored with diaminobenzidine (DAB, ZSGB-Bio, ZLI-9031, 1 : 100) and then counterstained with hematoxylin for 5 minutes [10]. The sections were observed under a microscope (Carl Zeiss Jena, Germany). Image-Pro Plus 6.0 image analysis system (Media Cybernetics, USA) was used to analyze, and 8 nonoverlapping fields of view were randomly read from each slice. The integrated optical density (IOD) was calculated and was taken for statistical analysis.

### 2.4. Statistical Analysis

Statistical analyses were performed with the Statistical Package for the Social Sciences, version 22.0 (SPSS Inc., Chicago, IL, USA). All data were described as mean ± standard deviation ($\bar{X}\pm s$) values. Differences between groups were analyzed by one-way analysis of variance (ANOVA), followed by Student-Newman-Keuls test. *P* values of less than 0.05 were considered to be statistically significant.

## 3. Results

### 3.1. Renal Hemodynamics of Rats

Renal ultrasonography of rats showed no significant difference in renal size among groups. However, compared with the WKY group, the vascular resistance index in the SHR group was higher (*P* < 0.05), and each treatment significantly decreased the vascular resistance index (*P* < 0.05, Figure 1). The valsartan group and the RA+RS group obviously decreased (Table 1). We speculate that these two drugs may reduce renal blood flow resistance and protect renal function in clinical treatment.

### 3.2. Biomarkers of Serum Renal Damage in Rats

The serum levels of NE, E, BNP, and Ang II were all increased in the SHR group than in the WKY group (*P* < 0.05). In addition, the RS group has decreased levels of E and BNP than the SHR group (*P* < 0.05), and the RA group has decreased NE, E, and BNP levels (*P* < 0.05). Simultaneously, the valsartan group had obviously reduced levels of NE, E, BNP, and Ang II (*P* < 0.05), and the herb pair of RA and RS obviously decreased the levels of NE, E, BNP, and Ang II (*P* < 0.05, Table 2).

### 3.3. Rat Renal Morphology

Compared with that in the WKY group, the density of AT1 and TGF-*β*1 was increased in the SHR group, and the density of NO was significantly decreased. After 4-week different drug administration, compared with the SHR group, all the treatment groups had decreased AT1 and TGF-*β*1 density, and the density of NO was increased (Figure 2). Compared with the WKY group, transmission electron microscopy showed that the SHR group had irregular cell morphology, endothelial cytoplasmic swelling, foot process fusion and foot process wide, organelle-rich, both atrophy of renal tubules, decreased cytoplasm, and thicker and crinkled basement membrane. Compared with the SHR group, after the drug treatment, all the groups have improved cell morphology, endothelial cytoplasmic swelling decreased, occasional fusion of foot process segmental fusion and neatly arranged, and the organelles were abundant (Figure 3). Among them, RA+RS proved to have the best efficacy.

## 4. Discussion

TCM has received extensive attention and research due to its long-lasting efficacy and fewer side effects [11]. TCM not only pays attention to improving the symptoms of patients but also focuses on the adjustment of the patients' constitution and improve the quality of life [12]. HRD is usually related to the insufficiency of “qi” and “blood.” Studies showed that RA can improve cardiovascular function and increase coronary blood flow [13, 14]. Simultaneously, treatment with RA may improve TGF-*β*1-induced renal fibrosis [15]. Studies reveal that RS can improve vascular function and structure and significantly improve the occurrence of hypertension [16], and RS and its extracts have been known to have an antioxidant property and neuroprotective effects [17]. The combination of RA and RS exerts synergistic effect on HRD.

Renal interstitial fibrosis (RIF) is the main pathological change from a variety of chronic kidney disease to end-stage renal disease [18]. Studies have found that for chronic kidney disease, tubulointerstitial damage is more important than glomerular disease [19]. Inhibiting epithelial-mesenchymal transition of renal tubular epithelial cells is considered an efficient approach for the treatment of renal interstitial fibrosis [20–22]. Currently, mechanisms of HRD have been paid more attention, such as hyperactivation of the renin-angiotensin system (RAS), small vessel lesions, and an increase in sodium and water retention. The kidney is densely innervated by sympathetic nerves, which are playing an important role in the regulation of blood pressure homeostasis [23]. Therefore, we discuss the mechanism of renal sympathetic nerve in HRD.

The main components of RAS such as Ang I and Ang II can be detected in normal human kidneys. Studies have found that aberrant RAS activation is closely related to RIF [24]. On the one hand, with the combination of Ang II and AT1 receptor, abnormal expression of Ang II can directly stimulate TGF-*β*1 activity and directly regulate the synthesis and degradation of extracellular matrix (ECM), regulating inflammatory mediators in the kidney and aggravating RIF [25, 26]. The second is that Ang II can activate signal pathways by stimulating the RAS system, which can induce cell proliferation and aggravate RIF. In our study, the combination of RA and RS obviously decreased the levels of BNP and Ang II. It is speculated that RA and RS can effectively reduce the expression of Ang II, block RAS activation and inhibit TGF-*β*1 expression, delay the progression of the RIF, and prevent hypertension and cardiac function injury (Figure 4).

Meanwhile, studies found that due to the decrease in renal vascular flow, stimulation of renal sympathetic nerves can cause hypertension [27]. Stimulation signals such as ischemia, hypoxia, and NO can activate the receptors of the renal sympathetic afferent nerves and transmission to the central nervous system [28, 29] and increase central sympathetic nerve activity by activating neurons in the rostral ventrolateral medulla, causing vasoconstriction and increased blood pressure [30, 31]. At present, changes in plasma noradrenaline concentration are used as an evaluation index of sympathetic nerve activity [32]. In our study, we found that NE and E in the SHR group were significantly increased; it suggests that there is sympathetic hyperexcitability in HRD. And the combination of RA and RS obviously decreased the levels of NE and E. It is speculated that RA+RS can effectively inhibit the overexcited sympathetic nerve in HRD.

The sympathetic nervous system regulates blood pressure and heart and kidney functions by releasing catecholamines. Simultaneously, the sympathetic nervous system can activate *β*1 receptors, leading to renin release and RAS activation. In addition, Ang II can promote the release of catecholamines, increase sympathetic nerve activity, and participate in the pathophysiological process of HRD [33].

In addition, this study still has limitations. The components of RA and RS are complex, and it is impossible to determine which specific active ingredients have played a role. The investigation of the pharmacological mechanism cannot be very clear. The follow-up research needs to be further verified.

In conclusion, the results of the present study suggested sympathetic overexpression in the pathogenesis of HRD. The combination of RA and RS may inhibit the hyperexcitability of sympathetic nerves, reduce Ang II overexpression, avoid abnormal activation of the RAS system, and improve rat renal blood flow resistance, accordingly maintaining the normal physiological structure and function of kidney tissue and having a protective effect on the cardiovascular system. Moreover, further comprehensive studies are required to examine other possible mechanisms.

## Figures and Tables

**Figure 1:** Renal ultrasonography of rat vascular resistance index: (a) RA group; (b) RS group; (c) RA+RS group; (d) valsartan group; (e) SHR group; (f) WKY group.

**Figure 2:** AT1, NO, and TGF-*β*1 density in the kidney determined by IHC staining (×400). AT1: angiotensin type 1; NO: nitric oxide; TGF-*β*1: transforming growth factor-*β*1; RA: *Radix Astragali* treatment group; RS: *Radix Salvia Miltiorrhiza* treatment group; RA+RS: RA and RS combination treatment group; SHR: spontaneously hypertensive rat group; WKY: Wistar Kyoto rat group.

**Figure 3:** Renal sections were observed under a transmission electron microscope (×12000): (a) RA group; (b) RS group; (c) RA+RS group; (d) valsartan group; (e) SHR group; (f) WKY group.

**Figure 4:** Mechanism of sympathetic activation in HRD.

**Table 1:** The rat renal vascular resistance index.

Group	No.	Right renal	Left renal
RA group	6	0.65 ± 0.04^∗^	0.67 ± 0.06^∗^
RS group	6	0.62 ± 0.03^∗^	0.67 ± 0.10^∗^
RA+RS group	6	0.54 ± 0.04^∗^	0.54 ± 0.05^∗^
Valsartan group	6	0.54 ± 0.04^∗^	0.57 ± 0.07^∗^
SHR group	6	0.75 ± 0.02^△^	0.80 ± 0.02^△^
WKY group	6	0.51 ± 0.04	0.53 ± 0.03

No.: number; RA group: *Radix Astragali* treatment group; RS group: *Radix Salvia Miltiorrhiza* treatment group; RA+RS group: RA and RS combination treatment group; SHR group: spontaneously hypertensive rat group; WKY group: Wistar Kyoto rat group. Values are the mean ± SD. ^∗^*P* < 0.05 vs. the SHR group; ^△^*P* < 0.05 vs. the WKY group.

**Table 2:** Renal biomarkers in rat serum.

Group	NE	E	BNP	Ang II
RA group	11.84 ± 0.41^∗^	0.92 ± 0.20^∗^	200.68 ± 5.46^∗^	152.76 ± 5.50
RS group	12.98 ± 0.97	0.89 ± 0.12^∗^	193.30 ± 5.48^∗^	153.26 ± 7.54
RA+RS group	8.57 ± 0.42^∗^	0.68 ± 0.04^∗^	186.13 ± 7.86^∗^	126.36 ± 10.29^∗^
Valsartan group	11.52 ± 0.65^∗^	0.70 ± 0.11^∗^	191.90 ± 6.43^∗^	132.94 ± 9.14^∗^
SHRs group	14.04 ± 1.39	1.40 ± 0.34	219.75 ± 9.33	157.87 ± 4.70
WKY group	8.14 ± 1.01^∗^	0.60 ± 0.07^∗^	159.58 ± 7.22^∗^	115.58 ± 7.60^∗^

RA group: *Radix Astragali* treatment group; RS group: *Radix Salvia Miltiorrhiza* treatment group; RA+RS group: RA and RS combination treatment group; SHR group: spontaneously hypertensive rat group; WKY group: Wistar Kyoto rat group; NE: norepinephrine; E: epinephrine; Ang II: angiotensin II; BNP: B-type brain natriuretic peptide. Values are the mean ± SD. ^∗^*P* < 0.05 vs. the SHR group.

## Data Availability

All data included in this study are available upon request by contact with the corresponding author.
